RETRACTED

# Common Pathogens and Drug Resistance of Neonatal Pneumonia with New Multichannel Sensor

**DOI:** 10.1155/2022/2208636

**Published:** 2022-08-08

**Authors:** Xueping Dong, Peipei Zhou, Guannan Zhu

**Affiliations:** Department of Pediatrics, Xuzhou First People's Hospital, Xuzhou, Jiangsu, China

## Abstract

This study aimed to study the application value of a new multichannel sensor in pathogen detection and drug resistance analysis of neonatal pneumonia. 180 newborns with infectious pneumonia were selected, and a new multichannel piezoelectric sensor was constructed. The traditional Kirby–Bauer (K–B) method and the piezoelectric sensor were adopted to detect the pathogens and drug resistance in newborn samples, respectively. The results showed that the sensitivity and specificity under the K–B method (99.58% and 99.32%) and the multichannel piezoelectric sensor (99.43% and 94.29%) were not statistically different (*P* > 0.05). The detection time (17.25 h) of the K–B method was significantly longer than that (7.43 h) of the multichannel piezoelectric sensor (*P* < 0.05). From the results of pathogen detection, it was found that *Klebsiella pneumoniae* accounted for a relatively high proportion of 25.1%, followed by *Staphylococcus aureus* and *Haemophilus influenzae* of 13.4% and 12.33%, respectively. The resistance rate of the *Staphylococcus aureus* to vancomycin and rifampicin was as high as 100% and that to gentamicin, ciprofloxacin, and erythromycin reached more than 50%. In short, the new multichannel piezoelectric sensor had the high sensitivity and specificity for the pathogens' detection of neonatal pneumonia, and it required a shorter time. The pathogens were mostly Gram-negative bacteria, followed by Gram-positive bacteria and fungi. *Klebsiella pneumoniae*, *Staphylococcus aureus*, and *Haemophilus influenzae* were the main ones. The neonatal pneumonia pathogens had also strong drug resistance against vancomycin, rifampicin, chloramphenicol, meropenem, amikacin sulfate, chloramphenicol, and many other antibacterial drugs.

## 1. Introduction

Neonatal pneumonia is the most common serious respiratory disease in the neonatal period. It is characterized by diffuse lung lesions and atypical clinical manifestations. It is an infectious disease and is one of the main causes of neonatal deaths [1, 2]. Different from pneumonia in older children, neonatal pneumonia is often atypical, accompanied by coughing occasionally, and the body temperature may not rise. The main symptoms are empurpling around the lips, foaming at the mouth, dyspnea, malaise, and refusal of milk. There are differences in the early symptoms of aspiration pneumonia and infectious pneumonia. The central nervous system manifestations can occur when the aspiration pneumonia develops severe symptoms, including respiratory failure, emphysema, atelectasis, pulmonary arterial hypertension, and hypoxic-ischemic encephalopathy [3, 4]. Infectious pneumonia can be caused by bacteria, viruses, and chlamydia, and it can be acute or chronic. With hematogenous infections, jaundice, hepatosplenomegaly, meningitis, and other multisystem symptoms are the main symptoms. Some severe patients may experience dyspnea, apnea, three concave signs, and even heart failure. Neonates with weaker immune function are susceptible to pathogens. If the mother suffers from infectious diseases before delivery, the pathogens can cause fetal infection through the placenta, and its symptoms appear within 24 hours after delivery [5, 6]. In addition, neonates have short trachea and drier lumens and their cilia have poor ability to remove bacteria and dusts, so bacteria are easy to descend into the lungs. The differentiation of neonatal lung tissues is not perfect, the alveolus is less, and the lungs are rich with blood vessels relatively; so, the neonates are easy to suffer from congestion and inflammation [7, 8]. Common pathogens that can cause neonatal pneumonia include *Staphylococcus aureus*, group B hemolytic *Streptococcus*, *Pseudomonas aeruginosa*, *Listeria*, *Chlamydia*, and some anaerobic bacteria and viruses [9].

RETRACTED

The multichannel series piezoelectric sensor is a new biochemical analysis method that combines the high sensitivity of the piezoelectric sensor and the specificity of biological response. This analysis method uses a single strand of reactive nucleotides as a probe, so that it can identify the detection targets accurately and deliberately in an environment with multiple components. Then, the detection and recognition process is converted into an easy-to-analyze electrical signal through the transducer [10, 11]. Studies have found that the multichannel series piezoelectric sensor has a certain application value and research potential in microbiology, molecular biology, protein, and gene detection. [12, 13]. At present, the detection of pneumonia pathogens such as viral pneumonia can be performed to detect the nucleic acid of the viruses through the detection of virus antibodies, isolation of the virus, high-throughput sequencing, and reverse transcription-polymerase chain reaction method [14, 15]. However, this detection method has a low positive rate within one week after onset, and the detection has high requirements on various aspects such as operating environment and personnel quality; thus, it is difficult to be widely applied in routine laboratories [16].

RETRACTED

For the improvement of the detection efficiency and effectiveness of neonatal pneumonia pathogens, it was tried to design a new multichannel series piezoelectric sensor. With its high sensitivity and antibody specificity, it was used for the detection of microorganisms and antibodies. Thereby, the common pathogens and drug resistance of pneumonia were analyzed.

## 2. Materials and Methods

### 2.1. General Information and Grouping of Patients

180 neonates with infectious pneumonia were included, as they were admitted to XXX Hospital from September 2016 to November 2020. There were 89 boys and 91 girls. It had been approved by the XXX Medical Ethics Committee, and the family members of the neonates got to know the content and methods and agreed to sign the corresponding informed consent.

The inclusion criteria were formulated as follows. The neonates were diagnosed with pneumonia by clinical and pathological methods. They were aged between 5 and 30 days. Family members of the kids agreed to accept the sample collection plan.

With the exclusion criteria, the newborns that met the following conditions were excluded. The neonates were complicated with diseases of other systems or organs. The neonates had bronchial asthma or congenital bronchopulmonary dysplasia. Their general information was incomplete.

### 2.2. The Multichannel Piezoelectric Sensor

The multichannel series piezoelectric sensor was to connect the piezoelectric quartz crystal after being oscillated in the gas phase to a pair of platinum mesh conductivity electrodes in series. The platinum mesh conductivity electrodes had a more sensitive response to the conductivity and permittivity of the liquid medium [17, 18]. The quartz crystal was sealed in a gaseous environment to prevent the crystal from being corroded by the liquid, thereby improving the service life of the crystal effectively. The loss of surface acoustic waves was small in the gas environment, which improved the stability of the oscillation frequency greatly [17, 18].  Figure 1 shows the structure of the multichannel series piezoelectric sensor.

The oscillation frequency of the multichannel series piezoelectric sensor was related to the conductivity and permittivity of the liquid medium, and its resonance frequency *P* could be expressed as

(1) $$\begin{array}{c} P=P_{0}\left[1+\frac{\pi P_{0}C_{q}\left(2\pi \right)P_{0}C_{s}-YG}{G^{2}-2\pi P_{0}C_{0}GY+4\pi^{2}P_{0}2C_{s}\left(C_{0}+C_{s}\right)}-\pi P_{0}C_{q}R_{q}Y\right], \end{array}$$

(2) $$\begin{array}{c} F_{\text{0}}=\frac{1}{\left(2\pi \sqrt{L_{q}C_{q}}\right)}. \end{array}$$

In the above equation (1), *P* represents the resonance frequency, *C*_*q*_ represents the dynamic capacitance of the quartz crystal vibration, *R*_*q*_ is the dynamic resistance of the quartz crystal vibration, *C*_0_ represents the static capacitance of the quartz crystal vibration, and *Y* is the oscillator phase transfer parameter.

(3) $$\begin{array}{c} G_{S}=k\chi . \end{array}$$

In equation (3), *k* is the cell constant of the piezoelectric impedance sensor and *χ* is the conductivity of the liquid medium.

(4) $$\begin{array}{c} C_{\text{s}}=k\varepsilon +C_{p}. \end{array}$$

In equation (4), *ε* is the dielectric constant of the solution and *C*_*p*_ is the capacitance between the two wires connected to the electrode. Under the condition of ensuring the stability of other parameters, the dielectric constant and conductance of the liquid medium determined the frequency change [19]. The schematic diagram of the sensor circuit is shown in Figure 2.

RETRACTED

Figure 3 shows the loop of the multichannel series piezoelectric sensor. Only when the loop gain was 1 and the phase shift was 0, the piezoelectric sensor could run with a stable frequency.

### 2.3. Sample Collection and Testing

For the neonates diagnosed with infectious neonatal pneumonia, a sterile suction tube was inserted from their nostril to the lower end of the respiratory tract after their admission, and the sputum of the kids was collected to the sterile sampling tube by negative pressure suction. The entire sample collection process was completed in a sterile environment. The suspension of the collected samples was then prepared and was added to the broth mediums (2 g beef extract, 1 g yeast extract, double distilled water, magnesium sulfate, calcium chloride, sucrose, and nutrient solution). The culture bottle was inserted into the piezoelectric sensor tester and was incubated for 18 hours at a constant temperature. All frequency shift curves would be recorded by the computer linked to the piezoelectric sensor.

The doubling dilution method was adopted to prepare the cefoxitin solution with a concentration gradient of 0.5–8 *μ*g/mL. The broth culture solution, prepared sample suspension, and antibiotic solution were added to the sterile detection cell. The detection cell was then sealed and inserted into the thermostatic piezoelectric biosensor. All frequency curves were recorded.

### 2.4. Drug Susceptibility Testing

In the drug susceptibility test, the hydrolyzed casein agar plate was used to carry out the Kirby–Bauer (K–B) method. A paper sheet containing a quantitative antimicrobial drug was sticked on the agar plate that was inoculated with bacteria to be tested. The drug contained in the paper sheet would absorb the water in the agar, dissolve, and continue to diffuse to the area around the paper sheet. Thus, a decreasing concentration gradient was formed. The growth of the bacteria to be tested was inhibited within the inhibitory concentration range around the paper sheet, resulting in a transparent inhibition zone.

RETRACTED

A pure culture colony with similar morphology was picked from the agar plate, and the broth medium was inoculated. It was cultured at a constant temperature until the turbidity reached 0.5 McFarland units. After being taken out, the broth was added to adjust the concentration of the bacterial solution to 0.5 McFarland units, and the bacterial content was about (1-2) × 10^8^ cfu/mL.

A sterile cotton swab was put into the adjusted bacterial suspension, and the redundant bacterial suspension on the tube wall was squeezed out. The lines were drawn on the hydrolyzed casein agar plate to cover the entire agar surface. The plate was rotated 60° to draw lines for three times. The edge of the agar was smeared with the swab at the last time, and it was left at room temperature for 3–5 minutes.

A paper dispenser or sterile tweezers were used to take the drug sensitive test paper, which was then sticked on the surface of the plate. The paper was gently pressed with the tip of the tweezers to make it flat. The distance between each piece of paper was not less than 24 mm, and the distance between the center of the paper and the edge of the plate was not less than 15 mm.

After the paper plate was incubated at 35°C for 20 hours, the diameter of the inhibition zone was measured with a vernier caliper. Standard quality control strains of *Escherichia coli* (ATCC25922), standard strains of *Staphylococcus aureus* (ATCC25923), and standard strains of *Pseudomonas aeruginosa* (ATCC27853) were used for quality control of all identification reagents and antibiotic strips for drug sensitivity analysis.

### 2.5. Statistical Methods

The data were analyzed by SPSS 19.0. The measurement data was expressed by the mean ± standard deviation ($\bar{x}\pm s$), and the enumeration data were expressed by percentage (%). Pairwise comparisons were performed using analysis of variance. *P* < 0.05 indicated that the difference was statistically significant.

## 3. Results

### 3.1. Detection Effect of the Multichannel Piezoelectric Sensor

Figure 4 shows the detection results of clinical strains by the K–B method and the multichannel piezoelectric sensor. The test results of the cefoxitin tablet method were taken as the determination criteria. It could be observed that the sensitivity and specificity of the K–B method were 99.58% and 99.32%, respectively; while those of the multichannel piezoelectric sensor were 99.43% and 94.29%, respectively. There was no statistically significant difference in both the sensitivity and the specificity between the two detection methods (*P* > 0.05). Thus, the detection results of the multichannel piezoelectric sensor were reliable. The detection time of the K–B method was 17.25 h, which was significantly longer than that of the multichannel piezoelectric sensor (7.43 h) (*P* < 0.05).

RETRACTED

### 3.2. Results of Pathogen Detection

The sputum of newborn patients with neonatal pneumonia was collected and cultured for detection, and the results are shown in Figure 5. It was shown that the pathogens of neonatal pneumonia were mainly Gram-negative bacteria, followed by Gram-positive bacteria and fungi. Among them, *Klebsiella pneumoniae* accounted for a relatively high proportion of 25.1%. It was followed by *Staphylococcus aureus* and *Haemophilus influenzae*, accounting for 13.4% and 12.33%, respectively.

### 3.3. Drug Resistance of Gram-Positive Bacteria in the Pathogens

Figure 6 shows the analysis results of drug resistance of the major Gram-positive bacterium—*Staphylococcus aureus* among neonatal pneumonia pathogens. The drug resistances were analyzed of *Staphylococcus aureus* to ampicillin, gentamicin, vancomycin, penicillin, rifampicin, ciprofloxacin, tetracycline, erythromycin, and other antibacterial drugs. It was suggested that the resistance rates of *Staphylococcus aureus* to vancomycin and rifampicin were as high as 100% and those to gentamicin, ciprofloxacin, and erythromycin were over 50%.

### 3.4. Drug Resistance of Gram-Negative Bacteria in the Pathogens

Figure 7 shows the results of drug resistance of *Klebsiella pneumoniae*, the main Gram-negative bacterium among neonatal pneumonia pathogens. Its drug resistances to several antibacterial drugs were analyzed, including those to imipenem, aztreonam, ciprofloxacin, chloramphenicol, meropenem, ceftazidime, amikacin sulfate, and ampicillin. It was found that the resistance rates of *Klebsiella pneumoniae* to both chloramphenicol and meropenem were as high as 100%. It was followed by those to amikacin sulfate and ciprofloxacin, which was 95.8% and 93.45%, respectively.

### 3.5. Drug Resistance of Extended-Spectrum *β*-Lactamase-Positive Bacteria

Figure 8 shows the drug resistance results of extended-spectrum *β*-lactamase-positive bacteria among the pathogens of neonatal pneumonia. The resistance rates were analyzed of *Escherichia coli* and *Klebsiella pneumoniae* to the antibacterial drugs like gentamicin, amikacin sulfate, chloramphenicol, cefazolin, aztreonam, levofloxacin, and piperacillin. It was observed that the extended-spectrum *β*-lactamase-positive bacteria in the neonatal pneumonia pathogens had the extremely high drug resistance rate of 80% to amikacin sulfate and chloramphenicol. The drug resistance rates of *Escherichia coli* to both gentamicin and levofloxacin were more than 50%.

RETRACTED

## 4. Discussion

Neonatal pneumonia is prone to occur in 1-2 weeks after birth, and the pathogenetic condition is usually complex, which causes serious harm to neonates. Therefore, it is very important to implement early and efficient detection, diagnosis, and treatment [20,21]. In view of the wide detection range and high sensitivity of the multichannel series piezoelectric sensor in microbiology, molecular biology, protein, and gene detection, it was intended to apply the prepared sensor to pathogen detection of neonatal pneumonia [22]. Studies have found that the pathogens of neonatal pneumonia mainly include *Streptococcus pneumoniae* and group B hemolytic *streptococcus*, *Staphylococcus*, *Staphylococcus aureus*, *Influenza bacillus*, and *Escherichia coli*. Most of them are Gram-negative bacteria, which are more common in low birth weight infants. The onset time is earlier and the clinical features are diverse. The initial manifestations are not obvious, the coughing is less, the breathing movement is superficial, and no specificity can be discovered in the symptoms. In addition, kids may also manifest as listlessness or restlessness, low response, vomiting, and abnormal body temperature. [23]. Except for a variety of Gram-negative bacteria, some viruses (respiratory syncytial virus, adenovirus, influenza virus, and parainfluenza virus) and fungi can also lead to neonatal pneumonia. There are obvious differences in the birth weight of neonates with pneumonia caused by different pathogens. The birth weight of neonates with pneumonia caused by *Staphylococcus aureus* is the heaviest, and the birth weight of neonates with pneumonia caused by *Klebsiella pneumoniae* is the lowest. 13% of *Staphylococcus aureus* are resistant to oxacillin; more than 80% are sensitive to antibiotics such as compound sulfa, teicoplanin, and quinolones, and the sensitivity to gentamicin and clindamycin reaches 60–70% [24]. The sensitivity of *Enterobacter cloacae*, *Klebsiella pneumoniae*, and *Escherichia coli* to cephalosporin is less than 50% and that of *Escherichia coli* to thiamine enzyme inhibitors is above 80%. The sensitivity of *Enterobacter cloacae* and *Klebsiella pneumoniae* to amoxicillin-clavulanate potassium is 17% and 37%, respectively, and that of *Escherichia coli* and *Enterobacter cloacae* to imipenem is 100%.

It was shown from the detection results of the neonatal pneumonia pathogens using a multichannel series piezoelectric sensor that the sensitivity and specificity of the K–B method were 99.58% and 99.32%, respectively, and those of the multichannel piezoelectric sensor were 99.43% and 94.29%, respectively. No statistically significant difference was observed in the sensitivity and specificity of the two detection methods (*P* > 0.05). Therefore, the detection results of the multichannel piezoelectric sensor had reliability. The detection time of the K–B method lasted for 17.25 h, significantly longer than that of the multichannel piezoelectric sensor (7.43 h) (*P* < 0.05). It was indicated that the piezoelectric sensor had similar sensitivity and specificity to the commonly used K–B method, and the detection results were reliable. The detection time required by the traditional method was reduced to a certain extent under the K–B method, and its application value was high. The pathogen detection results suggested that the pathogens of neonatal pneumonia were mainly Gram-negative bacteria, followed by Gram-positive bacteria and fungi. *Klebsiella pneumoniae* accounted for 25.1%; besides that, *Staphylococcus aureus* and *Haemophilus influenzae* had the proportion of 13.4% and 12.33%, respectively. These were similar to the results of Xie et al. [25], indicating that the detection method was highly reliable. The results of drug resistance showed that different neonatal pneumonia pathogens had strong resistances to various antibacterial drugs like vancomycin, rifampicin, chloramphenicol, meropenem, amikacin sulfate, and chloramphenicol. Therefore, anti-infective drugs and therapeutic drugs should be selected rationally in the clinical treatment to prevent the drug resistance of pathogens from affecting the therapeutic effect on neonates.

RETRACTED

## 5. Conclusion

Cases with neonatal pneumonia diagnosed clinically and pathologically were selected. The traditional method and new multichannel series piezoelectric sensor were adopted to detect pathogens, whose drug resistances were also analyzed. It was found that the new multichannel piezoelectric sensor had the high sensitivity and specificity for the detection of neonatal pneumonia pathogens, and required time was relatively shorter. Gram-negative bacteria were the major pathogens observed, followed by Gram-positive bacteria and fungi. *Klebsiella pneumoniae*, *Staphylococcus aureus*, and *Haemophilus influenzae* were the main ones. These neonatal pneumonia pathogens had strong drug resistances against many great antibacterial drugs, such as vancomycin, rifampicin, chloramphenicol, meropenem, amikacin sulfate, and chloramphenicol. However, the sources of cases included were relatively concentrated, which might have a certain impact on the results. The cases included were less and less representative, so the improvement and optimization should be made in subsequent experiments, to further research the application value of the new multichannel sensor in neonatal pneumonia pathogen detection and drug resistance analysis. In short, a certain reference basis was provided for the early diagnosis and treatment of neonatal pneumonia.

RETRACTED

## Figures and Tables

**Figure 1:** Structure diagram of the multichannel sensor.

**Figure 2:** Schematic diagram of circuit of the multichannel sensor.

**Figure 3:** The loop of the multichannel piezoelectric sensor.

**Figure 4:** Detection effect of the multichannel piezoelectric sensor. ^*∗*^Significant difference compared to the K–B method (*P* < 0.05).

**Figure 5:** Detection results of pneumonia pathogens. (a) a–c represent Gram-negative bacteria, Gram-positive bacteria, and fungi, respectively. (b) a–h represent *Escherichia coli*, *Acinetobacter baumannii*, *Enterobacter cloacae*, *Klebsiella pneumoniae*, *Haemophilus influenzae*, *Streptococcus pneumoniae*, *Staphylococcus aureus*, and others, respectively.

**Figure 6:** Drug resistance of *Staphylococcus aureus*. a–h represent ampicillin, gentamicin, vancomycin, penicillin, rifampicin, ciprofloxacin, tetracycline, and erythromycin, respectively.

**Figure 7:** Drug resistance analysis of *Klebsiella pneumoniae*. a–h stood for imipenem, aztreonam, ciprofloxacin, chloramphenicol, meropenem, ceftazidime, amikacin sulfate, and ampicillin, respectively.

**Figure 8:** Drug resistance analysis of *Escherichia coli* and *Klebsiella pneumoniae*. (a) The results of *Escherichia coli*. (b) The results of *Klebsiella pneumoniae*. a–g indicate gentamicin, amikacin sulfate, chloramphenicol, cefazolin, aztreonam, levofloxacin, and piperacillin, respectively.

## Data Availability

The data used to support the findings of this study are available from the corresponding author upon request.
